# Integrated Evaluation of Financial Risk in Coal Industry Restructuring: A Model of Linear Regression and PCA

**DOI:** 10.1155/2022/2395633

**Published:** 2022-10-07

**Authors:** Xianping Yuan, Ziqiu Zhang

**Affiliations:** Xi'an University Science and Technology, Xi'an 710699, China

## Abstract

Aiming at the integrated evaluation problem of financial risk in coal industry restructuring, a model of linear regression and PCA is put forward. This paper studies the univariate correlation and multivariable mixed correlation between the main business income and the book value of fixed assets and nonfixed assets in the statements of coal listed companies and gives the correlation function between the variables by using a variety of univariate linear, univariate nonlinear, and binary linear regression methods. It also points out that the coal enterprises in China are basically in the stage of increasing scale income at the present stage and can continue to achieve rapid increase in profits through mergers and acquisitions and other expansion methods. At the same time, it is also concluded that nonfixed assets, namely, intangible assets and human capital, contribute more to the main business income of coal enterprises in China, which objectively proves the correctness of our thinking of developing knowledge economy.

## 1. Introduction

As the two main bodies of transaction completion, where are the reasonable boundaries of enterprises and markets? This is a question that has been raised and explored in the economic management theory and practice in recent decades [1–5]. In the actual operation of enterprises, on the one hand, chain enterprises are popular, and enterprises are constantly “slimming down,” replacing the potential operating costs of enterprises with market transactions. On the other hand, mergers and acquisitions have been staged again and again all over the world. Multinational companies have incorporated market transactions into their own operation track and replaced market transactions with intraorganizational transactions [6–8]. These seem to be two trains running in the opposite direction, but they are both running towards the destination of high profits [9, 10]. Some are inconceivable, but there is a logical necessity of its memory. The author believes that the essential difference between the two trains lies in the characteristics of the industry in which they operate. For some competitive industries, because the barriers to entry and exit are not high, the competition between enterprises is far greater than monopoly, and the enterprise scale is too large, which will artificially increase the sunk cost [11–14]. Therefore, in this type of industry, enterprises with relatively small sunk costs show more prominent competitive advantages, especially when there are systemic risks such as policy risk and price risk, and these small-scale enterprises may be more likely to win the competition. In the industrial field like the coal industry, the barriers to entry and exit of the industry have greatly increased due to the existence of a large number of special assets.

The specificity of assets is reflected in the following three aspects: first, the specificity of location; second, the specificity of material assets; and third, the specificity of human capital. Through horizontal M&A, the sunk cost of special assets can be “diluted” on a larger scale; however, vertical M&A can “internalize” the costs that are difficult to transfer due to asset specificity. Therefore, the coal industry is more suitable to expand the scale of a single enterprise by means of mergers and acquisitions, so as to reduce its production costs by replacing external market transactions with internal transactions. In the production process of coal enterprises, the existence of coal mining safety risks makes the investment in this industry also have its particularity; at the same time, in the rapid development of China's national economy, coal enterprises are severely affected by the supply and demand of coal. The reason is that their enterprise size is relatively small, and they lack the right to price. They need to expand to replace external market transactions with their internal transactions. So, is this substitution endless? According to modern enterprise property rights theory, the scale expansion of enterprises has boundaries. When the transaction cost of marginal market is equal to the transaction cost of marginal organization, the scale expansion of enterprises will stop [15–18]. In other words, when the market transaction costs saved by the enterprise expansion are just exhausted by the management costs increased by the enterprise expansion, the motivation of the enterprise expansion disappears. Therefore, the expansion of enterprises is not unlimited but has its inevitable boundaries.

Since the last century, the merger and reorganization of enterprises has become the midwife of the birth of many super large enterprises. In these industries with the nature of natural monopoly, the economic scale of enterprises is relatively high. Enterprises achieve the economic scale point through continuous expansion and indeed have more competitive advantages in the industry [19–21]. However, the problem is that mergers and acquisitions are not the only way for enterprises to expand. Why do enterprises not choose other strategies and only favor this strategy?

In China's coal industry, until now, the production concentration is still low compared with the international level. The low industrial concentration will certainly cause a short board effect on the improvement of the labor production efficiency and technical level of the whole industry. This has become the consensus of the government and the industry. From the perspective of payment of M & A, the payment mode of horizontal M&A in China's coal industry generally adopts the following two methods: if both are state-owned enterprises in the same administrative division, the administrative free transfer may be adopted; however, private small and medium-sized coal mines generally require cash settlement.

It can be seen from the relevant process of the development of China's coal industry in recent years. On the one hand, under the policy guidance and the motivation of the enterprises themselves to become bigger and stronger, the tide of coal enterprise mergers and acquisitions has developed from horizontal mergers and acquisitions within the industry to cross industry vertical mergers and acquisitions or diversified mergers and acquisitions, and the industry concentration has been optimized. With the expansion of the scale of coal enterprises and the continuous increase of business scope, it cannot be ignored that the internal operating costs of enterprises will inevitably increase. On the other hand, the external environment for the survival of coal enterprises has been constantly optimized. The coal and electricity prices have been merged. The thermal coal and coking coal futures with the price discovery function and risk prevention function have been listed for trading. Electronic trading platforms for various coal industrial products are also being established one after another. Large coal special trade fairs have emerged, and the road network and storage terminals of coal transportation are also increasingly improved. All these make the external transaction cost of coal enterprises lower.

In the face of these two favorable development directions at the same time, how do coal enterprises choose to continue to expand their scale through external mergers and acquisitions or to maintain the existing scale and make more use of the external market to obtain profits? At this stage, where is the boundary of the expansion of coal enterprises? This is the motivation of this paper.

## 2. Financial Crisis Index Definition and Data Preparation

To evaluate the financial security status of coal enterprise mergers and acquisitions, the following financial crisis index [22–25] of the related companies in the coal industry is established.

We evaluate the financial security status of mergers and acquisitions of listed coal companies with the following indexes:

(1) $$\begin{array}{c} W=\beta_{0}+\beta_{1}X_{1}+\beta_{2}X_{2}+\beta_{3}X_{3}+\beta_{4}X_{4}+\beta_{5}X_{5}+\beta_{6}X_{6}\text{,} \end{array}$$

where

(2) $$\begin{array}{c} X_{1}=\frac{main\;business\;income}{book\;value\;of\;total\;assets}\text{,}\\ X_{2}=\frac{total\;profit+financial\;expenses}{book\;value\;of\;total\;assets}\text{,}\\ X_{3}=\frac{free\;cash\;flow}{book\;value\;of\;total\;assets}\text{,}\\ X_{4}=\frac{the\;total\;market\;value\;of\;equity}{total\;liabilities}=\frac{value\;of\;outstanding\;share\;capital+Non\;tradable\;stock\;market\;value}{total\;liabilities}\text{,}\\ X_{5}=\frac{retained\;earnings}{Book\;value\;of\;total\;assets}=\frac{undistributed\;profit+surplus\;reserve}{Book\;value\;of\;total\;assets}\text{,}\\ X_{6}=\frac{total\;amount\;of\;external\;guarantees}{totalnetassets}\text{.} \end{array}$$

The above index is called the financial crisis index of listed companies in the coal industry, or W-score for short.

To determine the parameters *β*_0_, *β*_1_, and *β*_6_ in formula (1), linear regression calculation is required. The six independent variables in formula (1) can be calculated according to the financial statement data of listed companies. Financial crisis index W has no actual corresponding index in reality, so it is necessary to specify an alternative index [26–31]. After multiple weighing, the logistic function of the quick ratio is selected as the approximate alternative index of W, which is

(3) $$\begin{array}{c} \hat{W}=\frac{1}{1+\exp\;\left(-qucik\;assets/Current\;liabilities\right)}. \end{array}$$

We check the annual report data of 20 major listed companies in the coal industry in China, and calculate the values of each variable, and some of them are shown in Table 1.

Due to the small number of observable companies, any set of cross-sectional data cannot meet the requirements of large samples, and only panel data can be used for regression.

## 3. Least Squares Linear Regression with W-Exponentials

According to the definition of the W-index, the independent variable and the surrogate index of the dependent variable are relative indicators, and the difference between their respective means is basically within an order of magnitude. We try to first perform an ordinary least squares linear regression (OLSLR) on the W-index.

We suppose the variables *x*_1_,…, *x*_6_, *w* satisfy the linear relationship [32–35]:

(4) $$\begin{array}{c} W=\beta_{0}+\beta_{1}X_{1}+\beta_{2}X_{2}+\beta_{3}X_{3}+\beta_{4}X_{4}+\beta_{5}X_{5}+\beta_{6}X_{6}+\varepsilon \text{,} \end{array}$$

where *β*_1_(*i*=0,1,…, 6) is a constant and *ε* is a random error. Each variable is observed *n* times, and the observed value is

(5) $$\begin{array}{c} X=\left(\begin{array}{ccc} x_{11} & \cdots & x_{16}\\ \vdots & \ddots & \vdots \\ x_{n1} & \cdots & x_{n6} \end{array}\right)\text{,}\\ W={\left(w_{1},w_{2},\ldots \ldots ,w_{n}\right)}^{\prime }\text{,} \end{array}$$

where *x*_*ij*_ represents the ith observation of variable *x*_*j*_.

The above data are equivalent to the scatter set *S*={(*x*_*i*1_,…, *x*_*i*6_, *w*_*i*_) | *i* ∈ (1,…, *n*)}. The estimated binary linear regression equation [36, 37] based on the above-observed data is

(6) $$\begin{array}{c} \hat{w}={\hat{\beta }}_{0}+{\hat{\beta }}_{1}x_{1}+\ldots +{\hat{\beta }}_{6}x_{6}\text{.} \end{array}$$

By

(7) $$\begin{array}{c} W=\left(1,X\right)B+E\text{.} \end{array}$$

We get

(8) $$\begin{array}{c} \hat{B}={\left({\left(1,X\right)}^{\prime }\left(1,X\right)\right)}^{-1}{\left(1,X\right)}^{\prime }W, \end{array}$$

where

(9) $$\begin{array}{c} B={\left(\beta_{0},\beta_{1},\ldots ,\beta_{6}\right)}^{\prime }E={\left(\varepsilon_{1},\ldots ,\varepsilon_{n}\right)}^{\prime }\hat{B}={\left({\hat{\beta }}_{0},{\hat{\beta }}_{1},\ldots ,{\hat{\beta }}_{6}\right)}^{\prime }\text{.} \end{array}$$

The regression result is

(10) $$\begin{array}{c} \hat{B}=\left(\begin{array}{c} 0.5287\\ -0.0452\\ 0.1531\\ 0.6633\\ 0.0061\\ -0.0259\\ -0.0258 \end{array}\right). \end{array}$$

Based on this regression result, the W-index can be expressed as

(11) $$\begin{array}{c} W_{OLS}=0.5287-0.0452X_{1}+0.1531X_{2}+0.6633X_{3}+0.0061X_{4}-0.0259X_{5}-0.0258X_{6}\text{.} \end{array}$$

Given a significance level of *p* = 0.05, we make an interval estimate of each parameter in B with a confidence level of 1-p = 95%. Each confidence interval is shown in Table 2:

We find the residual *r* of all 171 samples, and the residual of the regression result of the nth sample can be calculated by the following formula:

(12) $$\begin{array}{c} r_{n}=w_{n}-{\hat{w}}_{n}=w_{n}-\left({\hat{\beta }}_{0}+{\hat{\beta }}_{1}x_{n1}+\ldots +{\hat{\beta }}_{6}x_{n6}\right)\text{.} \end{array}$$

The residuals and the confidence intervals of the significance level *p* = 0.05 of the residuals are shown in Table 3:

The accuracy of the least squares regression is not high to ensure the confidence level of the regression, and it is necessary to allow a large confidence interval for the regression residuals. Of the 171 samples, there are still nine samples whose regression residuals are outside the confidence range.

To measure the fitting degree of the regression equation and the sample data, the coefficient of determination of the regression is calculated, and the formula is

(13) $$\begin{array}{c} r^{2}=\frac{SSR}{SST}=\frac{SSR}{SSR+SSE}\text{.} \end{array}$$

Among them, SSR is the regression sum of squares, and its formula is

(14) $$\begin{array}{c} SSR=\sum {\left(\hat{w}-\overset{‾}{w}\right)}^{2}\text{.} \end{array}$$

SST is the sum of squares of the total variance, and its formula is

(15) $$\begin{array}{c} SST=\sum {\left(w-\overset{‾}{w}\right)}^{2}\text{.} \end{array}$$

SSE is the sum of residual squares, and its formula is

(16) $$\begin{array}{c} SST=\sum {\left(w-\hat{w}\right)}^{2}\text{.} \end{array}$$

After calculating, the coefficient of determination of the least squares regression is

(17) $$\begin{array}{c} r^{2}=0.7232\text{.} \end{array}$$

It shows that the results of least squares regression can explain 72.32% of the total variation of sample data.

The significance test of the linear relationship between independent variables and dependent variables was carried out, and the specific steps were as follows:

Step 1: Make a hypothesis:
*H*_0_: The linear relationship is not significant.
Step 2: Specify the test statistic:
  (18) $$\begin{array}{c} F=\frac{SSR/1}{SSE/\left(n-6-1\right)}\text{.} \end{array}$$
It can be proved that when the null hypothesis H0 is established, the statistic F obeys the F distribution, then the first degree of freedom is 1, and the second degree of freedom is 171 − 9=162, that is, *F* ~ *F*(1,162).
Calculate
  (19) $$\begin{array}{c} F=68.3358\text{.} \end{array}$$
Step 3: Specify the significance level *p* = 0.05, check the F distribution table according to the two degrees of freedom, and find *F*_0.05_(1,120)=3.92.
Step 4: Make a decisionbecause
  (20) $$\begin{array}{c} F\gg F_{0.05}\left(1,120\right)>F_{0.05}\left(1,162\right)\text{.} \end{array}$$
*H*_0_ is rejected, and the linear relationship between the dependent variable and the independent variable is considered to be significant.
Further, the estimated standard error is calculated to measure the fitting degree of the least squares regression, and its formula is
  (21) $$\begin{array}{c} s_{w}=\sqrt{\frac{\sum {\left(w-\hat{w}\right)}^{2}}{171-8-1}}\text{.} \end{array}$$
After being calculated,
  (22) $$\begin{array}{c} s_{w}=0.0423\text{.} \end{array}$$
Calculate the standard deviation of the variable *w* for all samples as
  (23) $$\begin{array}{c} s=\sqrt{\frac{\sum {\left(w-\overset{‾}{w}\right)}^{2}}{167-1}}=0.0778\text{.} \end{array}$$
According to the value of *s*_*w*_ and *s*, the fitting degree of least squares regression is considered acceptable.

## 4. Principal Component Linear Regression for W-Index

The simple linear regression results of the W-index in the previous section are not very satisfactory [38, 39]. It is suspected that there is a linear relationship between the six independent variables. The correlation coefficient matrix of the six independent variables is calculated as follows:

(24) $$\begin{array}{c} corrcoef\left(X\right)=\begin{array}{cccccc} 1.0000 & 0.1614 & 0.2440 & 0.0782 & 0.2710 & -0.0903,\\ 0.1614 & 1.0000 & 0.5648 & 0.3007 & 0.6385 & -0.1919,\\ 0.2440 & 0.5648 & 1.0000 & 0.2457 & 0.2758 & -0.2724,\\ 0.0782 & 0.3007 & 0.2457 & 1.0000 & 0.3042 & -0.1591,\\ 0.2710 & 0.6385 & 0.2758 & \;0.3042 & 1.0000 & 0.0024,\\ -0.0903 & -0.1919 & -0.2724 & -0.1591 & 0.0024 & 1.0000. \end{array} \end{array}$$

Observing the above matrix, corrcoef(*X*_2_, *X*_3_)=0.5648, corrcoef(*X*_2_, *X*_5_)=0.6385, and it can be seen that there are obvious correlations between *X*_2_ and *X*_3_, and between *X*_2_ and *X*_5_.

The above corrcoef(*∗*) represents the operation of finding the correlation coefficient matrix between the matrix column vectors.

Principal component analysis is performed on the observed value matrix *X* of each variable, and the steps are as follows:

Step 1: Normalize the respective variables. If *X*_*n*_^0^ is a column vector, mean  (*X*_*n*_^0^) is the mean of *X*_*n*_^0^, and std  (*X*_*n*_^0^) is the standard deviation of *X*_*n*_^0^, and the normalized vector of *X*_*n*_^0^ is
  (25) $$\begin{array}{c} X_{n}^{1}=\frac{X_{n}^{0}-mean\;\left(X_{n}^{0}\right)}{std\;\left(X_{n}^{0}\right)}\text{.} \end{array}$$
Assuming that each column vector in *X* has been normalized above, the normalized observation matrix of independent variables is expressed as *X*^1^.
Step 2: Use Matlab software to perform principal component analysis on X1, and the program statement and results are as follows:
  (26) $$\begin{array}{c} \left[\text{pc},\text{score},\text{latent},t\text{square}\right]=\text{princomp}\left(X\right)\text{.} \end{array}$$
Principal component coefficient is obtained as
  (27) $$\begin{array}{c} pc=\begin{array}{ccccccc} 0.2744 & -0.1326 & 0.8421 & -0.4081 & -0.0379 & 0.1730 & 0.5497,\\ -0.1153 & -0.1590 & 0.3711 & 0.1112 & 0.7136 & 0.4726 & 0.2450,\\ 0.1025 & 0.3500 & -0.6624 & -0.3805 & 0.3486 & 0.0622 & -0.4932,\\ -0.7552 & -0.2391 & 0.0617 & 0.4761 & -0.4713 & -0.0782 & 0.0322,\\ 0.4880 & -0.5531 & -0.2258 & -0.8265 & -0.0751 & 0.0422 & -0.5021,\\ & & & 0.0800. & & & \end{array} \end{array}$$
The variance contribution rate of the principal components also can be obtained.
Eigenvalues of the covariance matrix are
  (28) $$\begin{array}{c} \text{latent}=\begin{array}{c} 2.3895,\\ 1.0516,\\ 0.9384,\\ 0.7752,\\ 0.6003,\\ 0.2474. \end{array} \end{array}$$
The cumulative contribution rate of the first four principal components is
  (29) $$\begin{array}{c} \frac{2.3895+1.0516+0.9384+0.7752}{2.3895+1.0516+0.9384+0.7752+0.6003+0.2474}=0.8587\text{.} \end{array}$$
That is, the first four principal components can explain 85.87% of the variance.
The first four principal components can be expressed as
  (30) $$\begin{array}{c} y_{1}=0.2741x_{1}^{1}+0.5499x_{2}^{1}+0.4726x_{3}^{1}+0.3482x_{4}^{1}+0.4762x_{5}^{1}-0.2255x_{6,}^{1}\\ y_{2}=-0.1322x_{1}^{1}-0.1153x_{2}^{1}+0.2453x_{3}^{1}+0.0625x_{4}^{1}-0.4715x_{5}^{1}-0.8265x_{6}^{1}\text{,}\\ y_{3}=0.8423x_{1}^{1}-0.1595x_{2}^{1}+0.1025x_{3}^{1}-0.4932x_{4}^{1}-0.0782x_{5}^{1}-0.0752x_{6,}^{1}\\ y_{4}=-0.4085x_{1}^{1}+0.3715x_{2}^{1}+0.3505x_{3}^{1}-0.7552x_{4}^{1}+0.0322x_{5}^{1}+0.0425x_{6}^{1}\text{.} \end{array}$$
Step 3: Perform a least squares linear regression on W based on variables *y*_1_ ~ *y*_4_.
Generate a matrix of principal component vectors as
  (31) $$\begin{array}{c} F=X1*pc\text{.} \end{array}$$
Regression with the first four principal components is given as
  (32) $$\begin{array}{c} \left[b,bint,r,rint,\text{stats}\right]=\text{regress}\left(W,\left[\text{ones}\left(171,1\right),F\left(1:4\right)\right],0.05\right)\text{.} \end{array}$$
The result is
  (33) $$\begin{array}{c} b=\begin{array}{c} 0.6247,\\ 0.0305,\\ 0.0236,\\ -0.0181,\\ 0.0190. \end{array} \end{array}$$
That is, the regression equation is
  (34) $$\begin{array}{c} w=0.6247+0.0305y_{1}+0.0236y_{2}-0.0181y_{3}+0.0190y_{4}+\varepsilon \text{.} \end{array}$$
Step 4: Form transformation of regression equation.
Convert this result to a regression form concerning variables *x*_1_^1^ ~ *x*_6_^1^:
  (35) $$\begin{array}{c} pc\left(:,1:4\right)*{\left[0.0316\;0.0217-0.0162\;0.0166\right]}^{\prime }\\ ans=\begin{array}{c} -0.0243,\\ -0.0131,\\ 0.0226,\\ 0.0266,\\ 0.0066,\\ 0.0090. \end{array} \end{array}$$
That is, the regression equation is
  (36) $$\begin{array}{c} \begin{array}{c} w=0.6247-0.0131x_{1}^{1}+0.0226x_{2}^{1}+0.0266x_{3}^{1}\\ +0.0066x_{4}^{1}+0.0090x_{5}^{1}-0.0243x_{6}^{1}+\varepsilon . \end{array} \end{array}$$
Further, convert the above results into regression for relative to variables *x*_1_ ~ *x*_6_:
  (37) $$\begin{array}{c} \begin{array}{c} \text{pc}\left(:,1:4\right)*\frac{{\left[0.0314\;0.0216-0.0167\;0.0162\right]}^{\prime }}{{\left(stdX\right)}^{\prime }}\\ ans=\begin{array}{c} -0.0406,\\ 0.3459,\\ 0.3040,\\ 0.0017,\\ 0.0484,\\ -0.1198, \end{array}\\ 0.6247-sum\left(pc{\left(:,1:4\right)}^{*}\frac{{\left[0.0314\;0.0216-0.0167\;0.0162\right]}^{\prime }}{{\left(st\;dX\right)}^{\prime }\cdot *{\left(meanX\right)}^{\prime }}\right),\\ ans=0.5569. \end{array}\text{.} \end{array}$$
That is, the regression equation is
  (38) $$\begin{array}{c} \begin{array}{c} w=0.5569-0.0406x_{1}+0.3459x_{2}+0.3040x_{3}\\ +0.0017x_{4}+0.0484x_{5}-0.1198x_{6}. \end{array} \end{array}$$
Based on this regression result, the W-index can be expressed as
  (39) $$\begin{array}{c} \begin{array}{c} W_{PCA}=0.5578-0.0427X_{1}+0.3472X_{2}\\ +0.3019X_{3}+0.0030X_{4}+0.0463X_{5}-0.1185X_{6}. \end{array} \end{array}$$
Step 5: Analysis of regression results is done.
The determination of regression coefficient is
  (40) $$\begin{array}{c} r^{2}=0.5754\text{.} \end{array}$$
It shows that the results of principal component regression can explain 57.54% of the total variation of the sample data.
The linear relationship [39–41] between the independent variable and the dependent variable is tested for significance, and the calculation can be obtained as
  (41) $$\begin{array}{c} F=54.8235\text{.} \end{array}$$
We specify a significance level of *p* = 0.05 because *F* ≫ *F*_0.05_(1,120) > *F*_0.05_(1,162) rejects H and believes that the linear relationship between the dependent and independent variables is significant.
Further, the estimated standard error is calculated to measure the degree of fitness of the least squares regression, and after calculation, we get
  (42) $$\begin{array}{c} s_{w}=0.0522\text{.} \end{array}$$

From the above results, it can be seen that in this case, the regression determination coefficient of the principal component regression method is less than that of the least squares regression. The estimated standard error of the principal component regression method is larger than that of the least squares regression. Therefore, it is judged that the regression quality of the principal component regression method is worse than that of the least squares regression method in this example.

## 5. Discussions

Financial crisis and financial security are two different expressions of the same problem in a sense. Generally speaking, a company's high level of financial security is equivalent to its low level of crisis, and vice versa. Although the research on “financial security” and “financial crisis” has some subtle differences in emphasis, the two focus on the same goal on the whole. We make statistical analysis on the financial crisis of enterprises by using a large number of financial data and then draw statistical judgment and prediction. Generally, the following ideas are available:

  Make statistical analysis on the enterprises that have produced financial crisis, find their commonness, and establish a certain measure of financial crisis–crisis index
  The enterprises in financial crisis and financial security are matched and observed, and the variation information is obtained by comparing the indicators or indicators, and the variation information is analyzed to establish a measure of the degree of financial crisis

The above two methods are meaningful in theory, but in practice, the effect is not ideal. The reasons are as follows.

For the first method, the number of enterprises in financial crisis is not large, and it is difficult to obtain large samples with a statistical value. In addition to simple financial problems, there are many complex reasons leading to the financial crisis, which makes the overall situation of enterprises in the financial crisis very poor. It is difficult to draw a conclusion with strong causality by simply studying financial data. Thirdly, “financial crisis” is a kind of unstable state. The random fluctuation of financial data of enterprises in financial crisis state is more severe, and it is more difficult to have a statistical conclusion with a high confidence level.

For the second method, firstly, the selection of matching enterprises with enterprises in crisis is subjective, which will introduce uncontrollable systematic errors to the research results. Secondly, it is difficult to extract the crisis variation information objectively and effectively. Generally speaking, it is relatively objective to give a binary evaluation of 0 or 1 to a certain financial index of a paired enterprise, but the statistical processing of random variables with multidimensional 0–1 distribution requires very large statistical samples, which is impossible to achieve. If the nonbinary crisis variation data are processed, when selecting different matching enterprises, the crisis variation data extracted from the same crisis enterprise may be very different. In a sense, the research effect of the second method depends more on the “sense” of the researcher or the “smell” of the crisis.

In order to make the research results more objective, the following third method is adopted in this paper: Carry out statistical analysis on the financial data of enterprises in the financial security or “generally safe” state, establish a certain measure of financial crisis degree—crisis index, observe the financial data of a certain number of enterprises in the crisis state, calculate the observed value of crisis index, make necessary adjustments to the parameters of crisis index according to the observed value, and determine the value range of various financial states on the crisis index.

In a sense, the W-index established in this paper is actually a measure of the degree of “financial security,” and the degree of financial crisis can be derived from the degree of financial security. Since the financial data of enterprises in financial security are generally safe have strong commonality, the objectivity and confidence of W-index can be guaranteed.

The financial crisis index W, as a supplementary correction result to the Z-value discrimination model not only retains the original advantages of the Z-value discrimination model, which are easy to operate and intuitive, but also can give reasonable consideration to the contingent risks of the guaranteed liabilities when the enterprise provides guarantee to all subsidiaries or branches within the group or guarantee to other enterprises outside the enterprise. At the same time, the original judgment standard value in the Z-value judgment model is replaced by the mathematical treatment of “quick ratio” which is more practical and widely used. These two amendments and supplements make up for the defect that the Z-value discrimination model does not consider the off balance sheet business risks.

When the multivariate linear discriminant model calculates the value of *Z* by weighting and summarizing five financial indicators to predict the financial crisis, the off balance sheet business was not common in the enterprise financing business at that time. However, in the financial financing activities of large enterprises in China (especially those with state-owned background), the guarantee business is very common, and some enterprises even cross guarantee each other. In this way, once any one of the credit risk or liquidity risk occurs in a certain link of these debt chains, it may cause a chain reaction similar to the US financial crisis.

Therefore, it is of practical significance to introduce the financial crisis index W when evaluating the financing risk of M&A of coal enterprises in China. According to the above calculation results and the financial data of coal enterprises, the author believes that when *w* ≥ 0.55, the enterprise is relatively stable in terms of finance; when *w* < 0.5, the enterprise is in or will soon be in financial difficulties; and when 0.5 ≤ *w* ＜0.55, it belongs to the early warning zone. Such enterprises must make necessary intervention to the existing financial situation to prevent further deterioration of financial risk.

## 6. Conclusions

Until now, most of China's large coal enterprises have completed the signing of the main contract of merger and reorganization, but this does not mean the completion of the merger and reorganization task. This is because, on the one hand, the performance period of some contracts is relatively long and the restructuring payment has not been completed; on the other hand, the integration of merger and reorganization has a long way to go, especially in the current situation where the contradiction between supply and demand in the coal market is prominent and the coal price continues to decline, and the success of the reorganization and integration is more important. So how to determine which enterprises' financial situation is in a safe critical point in the short term? Considering that in the process of M&A financing of coal enterprises in China, a large number of “guaranteed loans” are used to finance from banks, and the phenomenon of mutual guarantee and cross guarantee among coal enterprises is serious, and these data are not reflected in the enterprise's balance sheet and not included in the previous commonly used financial risk evaluation indicators.

On the basis of Z-index, this paper adds the risk evaluation factor of enterprise's external guarantee, modifies the original risk judgment standard, puts forward the W-index to evaluate the financial risk of coal enterprise's M&A financing, and determines the parameters of W-index by regression analysis with three methods. Using three methods to calculate the previous financial data of some coal listed companies in China, the W-index value is obtained. According to the above calculation results and the financial data of coal enterprises, the judgment interval of W-index value is deduced; that is, when *w* ≥ 0.55, the enterprise is relatively stable in terms of finance; when *w* < 0.5, the enterprise is in or will soon be in financial difficulties; and when 0.5 ≤ *w* ＜0.55, it belongs to the early warning zone. Such enterprises must make necessary intervention to the existing financial situation to prevent further deterioration of financial risk. By using the derived W-index calculation formula and the above three methods, the W-index of some coal listed companies in China in recent years is calculated, respectively. Through comprehensive analysis and judgment, several representative W-index values are selected to indicate the “financial distress” or “financial warning” of the enterprise and the year when the enterprise turns stable after the distress or warning, and the reliability of the W-index is verified by analyzing the annual report of the enterprise in that year. However, due to the limited scale data of the current coal enterprises, the inflection point of economic scale (the dividing point between increasing scale income and decreasing scale income) cannot be reached, and it needs to be further analyzed after the subsequent development data of the enterprises are increased.

## Figures and Tables

**Table 1:** Data for regression of W-score (part).

Listed company	Serial number	Years	**X**_1_ = sales/total assets	**X**_2_ = EBIT/total assets	**X**_3_ = working capital/total assets	**X**_4_ = total market value of equity/total liabilities	**X**_5_ = retained earnings/total assets	**X**_6_ = total external guarantees/total net assets	**W**
Company A	1	2001	0.6308	0.1354	0.1548	6.361	0.049	0	0.6606
	2	2002	0.5218	0.1258	0.1815	7.1257	0.0431	0	0.7748
	3	2003	0.5209	0.1689	0.1975	4.8741	0.0554	0	0.687
	4	2004	0.6255	0.3638	0.2058	3.2146	0.2182	0	0.7754
	5	2005	0.5055	0.2236	0.0681	1.3452	0.1607	0.0375	0.5485
	6	2006	0.4458	0.0828	0.019	0.7992	0.0716	0.3196	0.513
	7	2007	0.7455	0.0753	0.1215	2.0585	0.1021	0.5183	0.5653
	8	2008	0.7755	0.1268	0.1408	0.5222	0.143	1.0414	0.5612
	9	2009	0.5692	0.0713	0.0711	1.915	0.1299	1.2118	0.5352
	10	2010	0.6864	0.0886	0.0803	1.4073	0.1237	0.8612	0.5425
	11	2011	1.0194	0.0736	0.1066	0.6693	0.1059	0.5436	0.5466
	12	2012	0.7062	0.0349	0.0434	0.4316	0.0843	0.5709	0.5193

Company B	13	2004	1.0399	0.1913	0.2217	2.1185	0.2321	0	0.6224
	14	2005	1.0361	0.1927	0.1197	2.2878	0.2945	0	0.5844
	15	2006	1.0013	0.2272	0.3107	1.1938	0.305	0.0091	0.5829
	16	2007	0.9621	0.2158	0.1507	1.8247	0.2549	0.01	0.5364
	17	2008	1.2081	0.2234	0.1594	0.3759	0.4163	0.0029	0.5212
	18	2009	0.3273	0.0824	0.2047	0.9709	0.1309	0.0027	0.5989
	19	2010	0.593	0.1124	0.112	1.7664	0.1776	0.0017	0.578
	20	2011	0.6671	0.1167	0.1495	1.4662	0.2195	0	0.6069
	21	2012	0.6807	0.077	0.1142	1.9876	0.263	0.0015	0.5846

**Table 2:** Confidence interval of OLSLR.

Parameter	Confidence interval
*β*_0_	(0.5091, 0.5506)
*β*_1_	(−0.0642, −0.0261)
*β*_2_	(0.0096, 0.2957)
*β*_3_	(0.5637, 0.7638)
*β*_4_	(0.0035, 0.0085)
*β*_5_	(−0.0855, 0.0339)
*β*_6_	(−0.0638, 0.0061)

**Table 3:** Residuals and confidence intervals of OLSLR (part).

Order	Regression residuals	Confidence intervals for residuals
1	−0.0007	(−0.0814, 0.0791)
2	0.0879	(0.0088, 0.1674)
3	−0.0038	(−0.0844, 0.0761)
4	0.0679	(−0.0072, 0.1433)
5	−0.0401	(−0.1194, 0.0381)
6	−0.0162	(−0.0966, 0.0647)
7	−0.0178	(−0.0983, 0.0622)
8	−0.0156	(−0.0902, 0.0592)
9	−0.0004	(−0.0733, 0.0722)
10	−0.004	(−0.0817, 0.0739)
11	−0.0042	(−0.0843, 0.0752)
12	0.0027	(−0.0771, 0.0830)
13	−0.0434	(−0.1245, 0.0372)
14	−0.0132	(−0.0941, 0.0679)
15	−0.1417	(−0.2189, −0.0646)

## Data Availability

The dataset can be accessed upon request.
